# TCM-ISP: A Comprehensive Intelligent Service Platform for Industry Chain of Traditional Chinese Medicines

This article has been retracted.

**DOI:** 10.1155/2021/9938625

**Published:** 2021-05-04

**Authors:** Ting Ting Cao, Xian Rui Wang, Xu Wei Sheng Ji, Hui Wang, Yun Wang

**Affiliations:** Information Engineering Research Center for Traditional Chinese Medicine, Beijing University of Chinese Medicine, Beijing 102488, China

## Abstract

In order to promote information interaction, intelligent regulation, and scale management in Chinese medicines industry, in this paper, a Chinese medicines intelligent service platform with characteristics of flexibility, versatility, and individuation was designed under the guidance of theoretical model of intelligent manufacturing of Chinese medicines (TMIM). TCM-ISP is a comprehensive intelligent service platform that can be flexibly applied to all links of Chinese medicines industry chain, which realizes data integration and real-time transmission as well as intelligent-flexible scheduling of equipment in response to different demand. The platform took logical framework of data flow as the core and adopts the modular design in which microcontroller and sensor module are independent to obtain overall design scheme of TCM-ISP that contains the diagram of overall framework, hardware structure, and software technology. Then, on the groundwork of overall design scheme and modern science technology, TCM-ISP was successfully constructed with flexible, intelligent, and networked characteristics in which TTL-USB and TTL-RS485S were utilized to build unified interface between boards with supporting hot-plugging mode. The results of platform tests show that TCM-ISP can not only successfully realize the integration, real-time transmission, and display of data information but also well accomplish remote intelligent-flexible control of equipment and allow flexible configuration and expansion of sensors and devices according to the needs of each link in TCM's industry chain. It is of great practical significance to the pursuit of intelligent manufacturing of Chinese medicines and the promotion of modernization of Chinese medicines industry.

## 1. Introduction

The Chinese medicines industry is gradually showing the modern development tendency of market demand-oriented, large-scale, and intelligent management mode [1, 2]. However, the modernization and upgrading of Chinese medicines industry are still slow due to many obstacle factors. Specifically, (1) cultivation of Chinese herbal medicines: the cultivation of Chinese herbs is mainly scattered planting, which is just managed by traditional experience, but also at primary stage of “living off the weather.” (2) Storage and processing of Chinese herbal medicines: the storage conditions for herbs are so rudimentary that quality cannot be guaranteed. From the perspective of herbal processing, the process and equipment are still in the semimechanized and mechanized production stage, making it difficult to keep up with the pace of times. (3) Discordance and low level of organization in the TCM industry chain: the uncoordinated development, low organization, and lack of linkage of various links of Chinese medicines industry chain have resulted in blocked information transfer and feedback and disconnection from market demand [3–5]. In a word, the low degree of informatization and intelligence of Chinese medicines industry and the backward management mode are the fundamental factors to restrict the modernization development of Chinese medicines industry.

In order to break above barriers and promote the modernization of the Chinese medicines industry, the following two works are indispensable. One is that information collection and real-time presentation of multiple aspects of Chinese medicines industry to provide reference for users and managers; the other is information integration processing and equipment intelligent scheduling in multiple aspects of Chinese medicines industry. To this end, in “Industry 4.0” era characterized by Internet to things (IOT) and information technology [6–9], a series of studies had been conducted. For example, the traceable system of cultivation process for Chinese herbal medicines (TSCM) was constructed on the basic of “Good Agricultural Practice (GAP)” and “Standard Operating Procedure (SOP)” to realize the traceability of cultivation information and the monitoring information, which has significant implications for intelligent control of Chinese medicines cultivation industry [10]. In response to the current situation of gum production, Wang carried out the design of MES system to build an intelligent management platform for gums, which improved production intelligence [11]. As for stages of extraction, concentration, and recovery in the process of Chinese medicines, researchers developed the automatic intelligent control system, resulting in increased productivity [12]. Moreover, TCM information resource platform had been established to provide information inquiry and consulting services for an enterprise, or to provide academic exchange and results transformation services for scientific researchers [13, 14].

These researches brought convenience for Chinese medicines industry. There was no doubt that research results had contributed to the modernization development of Chinese medicines industry to certain extent. However, the above researches more either focused on a certain aspect or provided more single services such as query and communication service. Considering the about there were local and functional limitations, and an ideal platform should be able to serve users from multiple aspects, including on-site monitoring, information interaction, and equipment dispatching command. We remain lacking a comprehensive intelligent service platform for Chinese medicines industry. It is significant to establish a comprehensive intelligent service platform to realize real-time monitoring, information communication, and equipment intelligent scheduling in each link of TCM's industry chain for promoting the modernization of Chinese medicines industry.

In this paper, an easy-to-operate, highly scalable, comprehensive Chinese medicines intelligent service platform (TCM-ISP) was constructed on the basic of theoretical model of intelligent manufacturing of Chinese medicines (TMIM) with taking interaction of data as core and new generation of information technology as support. Under guidance of TMIM, the overall construction plan was obtained through the design of platform functions, logical framework of data flow, overall structural framework, and technology roadmap. According to overall construction plan, the construction of TCM-ISP was completed by taking advantage of modern science technology. The platform can not only be applied to each link of Chinese medicines industry chain but also realize the integration, interaction, and intelligent control of information, which is conducive to promoting the informationization, intelligence, and modernization of Chinese medicines industry.

As shown in Figure 1, the platform system consists of a service platform and a plurality of distributed monitoring points. Among platform systems, the platform base points include gateway nodes, database, and web server, at the same time, each monitoring point makes up of a sensor, an application device, an analog-to-digital conversion device, a microcontroller, and a wireless transmission module. Each monitoring point can not only process sensor data but also communicate with API of service platform. After registering and obtaining corresponding permissions, users can browse and count the information in the detected area remotely, irregularly, and in various ways to realize remote real-time monitoring and management. Back-end database is used for data storage and recall.

The process of building Chinese medicines intelligent service platform system was as follows: firstly, flexible, intelligent, and networked platform functions were designed on the premise of analyzing user needs based on the current situation of Chinese medicines industry. Secondly, under the guidance of TMIM, the data flow logic framework of Chinese medicines intelligent service system was constructed by using data transmission rules. Then, the overall structural framework of system, hardware structure diagram of monitoring point, and technology roadmap was designed on the basic of the above logic framework to obtain overall construction scheme. Finally, according to the overall construction scheme, using modern science technology to complete the platform construction.

## 2. Functional Structure Design of Chinese Medicines Intelligent Service Platform

On the groundwork of analyzing user needs based on the current situation of Chinese medicines industry, the platform aimed to provide a service window for ordinary users to view production situation of each link. It can also provide workers with services such as information integration, real-time display, historical inquiry, and flexible intelligent control of equipment in multiple aspects of industrial chain. The functional design of platform focused on structural systematization, versatility, and scalability. As shown in Figure 2, the functional framework was divided into five major functional modules, namely, user management, sensor management, detailed monitoring, application device control, and data processing.

### 2.1. User Management

User management module mainly provides users with functions such as registration, login, password retrieval, password modification, and permissions. The platform divided users into two categories: general users and administrators. The former can browse the services and user usage by registering and logging in TCM-ISP; at the same time, the latter can configure utilities, authorize users, set the global platform, and monitor nodes.

### 2.2. Sensor Management

TCM-ISP consists of a server side platform and a plurality of distributed monitoring points. Monitoring points can be equipped with a variety of sensors to collect real-time data in the deployment environment. Each monitoring point had a corresponding service application program to process data and communicated with platform through API. Various sensors will be used on the platform to meet normal functions, such as illumination sensors, air temperature and humidity sensors, soil temperature and humidity sensors, and flow-meter, pressure sensors [15, 16]. After logging into the platform, managers can flexibly configure monitoring points according to specific needs.

### 2.3. Detailed Monitoring

Monitoring details were mainly reflected on the data and equipment status display. The platform can present real-time monitoring data, historical data and device-operating status, and so on, which provide reference for users. The forms of data presented in the platform are line charts, data tables, and so on. It is worth noting that administrators have access to all monitoring data, while users can only see a portion of data due to the difference in permissions.

### 2.4. Device Management

The TCM-ISP provided device control and triggering functions. Control refers to an action that the user intends platform to perform automatically; meanwhile, trigger refers to a user-set trigger condition. If the actual situation meets the set trigger conditions, the defined actions were executed to achieve a flexible combination. The combination of control and trigger can realize real-time operation and intelligent self-regulation between devices.

### 2.5. Data Processing

This module mainly provided users with data processing services such as data storage, judgment, and arithmetic. Real-time monitoring data were stored in a back-end database for review. Through setting thresholds of different monitoring indicators or mathematical relationships, the application device will trigger to realize remote networked control when meeting the requirement.

## 3. Data Flow Logic Framework of Chinese Medicines Intelligent Service Platform

The logical framework of data flow is a means to describe the flow and processing of data in the system in a detailed and objective way, which is the basis for guiding the design of system solution. According to the information interaction and device intelligent management requirements, the realization of platform functions requires a detailed understanding of logical structure of data flow. Therefore, this paper constructed a logical framework for the data flow of Chinese medicines intelligent service platform (TCM-ISP), which was built on the basic of theoretical model of intelligent manufacturing of Chinese medicines (TMIM).

### 3.1. Theoretical Model of Intelligent Manufacturing of Traditional Chinese Medicines

TMIM aims to address the lack of theoretical guidance in development process of intelligent manufacturing of Chinese medicines. TMIM is an intelligent manufacturing paradigm with entity grammar system as its theoretical framework, which aims to guide the construction of intelligent systems and pursuits personalized customization and flexible combination of devices as well as networked information transmission [17].

#### 3.1.1. Entity Grammar System

Entity grammar system (EGS) is a formal grammar system established for modeling of complex systems [17, 18]. It has a general structure capable of expressing mathematical axiomatic. In entity grammar system, an entity is defined as *E*=(*V*, *F*) that represents collection of all *F*-entities for *A*, in which alphabet *V* represents a set of symbols and alphabet *F* represents a set of functions (or operations). Entity grammar system can be strictly described as follows:

 
*λ* ∈ *E*=(*V*, *f*), *λ* symbolizes null set with no characters;
 
*V*⊆*E*=(*V*, *f*);
 
*f*(*ξ*_1_,…, *ξ*_*n*_) ∈ *E*=(*V*, *f*) is available from all *f* ∈ *F*, along with all *ξ*_1_,…, *ξ*_*n*_ ∈ (*V*, *f*);
 
*E*^+^(*V*, *F*)=*E*(*V*, *F*) − {*λ*} is a nonempty set of *F*-entities for *V*;

If *f* is an *n*-ary operation in *F*, the set of positions of *f* is the set Pos(*ξ*)={1,2,3,…, *n*}. The set of positions of an entity *ξ*=*f*(*ξ*_1_,…, *ξ*_*n*_) ∈ *E*=(*V*, *f*), showed by Pos(*ξ*), can be expressed as follows:

 
Pos(*λ*)=Φ;
  For *ξ* ∈ *V*, Pos(*ξ*)={*λ*};
  For an entity *ξ*=*f*(*ξ*_1_,…, *ξ*_*n*_),
 
Pos(*ξ*)=∪_*i*=1_^*n*^{*ip|p* ∈ Pos(*ξ*_*i*_)}.
  The size |*ξ*| of an entity is the cardinality of Pos(*ξ*).

The entity is deemed as pseudo-*f*-entity in the case of one or more *ξ*_*i*_ which is *λ* in an entity that is expressed by *f*(*ξ*_1_,…, *ξ*_*n*_). In the same way, with regard to all operations *f* in *F*, the set of pseudo-*f*-entities is called pseudo-*F*-entities, which is denoted by PEE. If any set *A*⊆*E*(*V*, *F*), as well as *f*(*A*)=*A*, then operation *f*: (*E*(*V*, *F*))^*n*^⟶*E*(*V*, *F*) in *F* is referred to pseudo-operation.

A whole entity grammar system, denoted by alphabet *G*, is a quintuple, that is to say, *G*=(*V*_*N*_, *V*_*T*_, *F*, *P*, *S*), where *V*_*N*_, *V*_*T*_ represents the finite set of nonterminal characters and terminal symbols, respectively. There is relationship between *V*_*N*_ and *V*_*T*_ : *V*_*N*_ ∪ *V*_*T*_=*V*, *V*_*N*_∩*V*_*T*_=Φ.

*F* represents the finite set of operations: *F*={*f*_*i*_*|f*_*i*_ : (*E*(*V*, *F*))^*n*^⟶*E*(*V*, *F*),  1 ≤ *i* ≤ *m*,  *m*, *n* ∈ *N*}.

*P* is the inference rule of *α*⟶*B*, *α* ∈ *E*^+^(*V*, *F*), *β* ∈ *E*(*V*, *F*).

*S* marks initial state of the system.

Let *G*=(*V*_*N*_, *V*_*T*_, *F*, *P*, *S*) become an entity grammar with the following formula: *L*(*G*)={*ξ* ∈ *E*(*V*_*T*_, *F*)*|S*⟹_*G*_^*∗*^*ξ*}.

The set is “language” produced by entity grammar system, where *S*⟹_*G*_^*∗*^*ξ* refers to an unspecified number of derivations that can be taken from *S* to *ξ*. If *x*, *y* ∈ *E*(*V*, *F*) and *f* ∈ *F*, then *x*⟹*Gy*. We consider that *y* is directly ratiocinated from *x* in *G*. For inference, rule of *α*⟶*β* in *P* with *u*, *v* ∈ *E*(*V*, *F*), *x*=*f*(*u*, *α*, *v*) ,  and *y*=*f*(*u*, *β*, *v*).

If the difference between nonterminals and terminals is not considered, as a result, entity grammar system (EGS) can be expressed as *G*=(*V*, *F*, *P*, *S*).

### 3.2. Construction of Theoretical Model of Intelligent Manufacturing of Traditional Chinese Medicines

On the foundation of EGS, a quadruple *Q*=(*V*, *F*, *P*, *S*) can express the theoretical model of intelligent manufacturing of traditional Chinese medicines:

1. *V*=*V*_1_ ∪ *V*_2_, where *V* is a collection of symbols that make up an entity in the production process, *V*_1_ is the set of attributes of processing object and *V*_2_ is the set of device parameters.
2. $\begin{array}{c} F=F_{1}\cup F_{2}\cup F_{3},\\ F_{1}=k\left(f\left(x\right),g\left(y\right)\right),\;x\in V_{1},y\in V_{2},\\ F_{2}=f\left(x\right),\\ F_{3}=g\left(y\right). \end{array}$
3. $\begin{array}{c} P=P_{1}\cup P_{2}\cup P_{3},\\ P_{1}=\left\{f\left(x\right)\right\},P_{2}=\left\{g\left(y\right)\right\},\\ P_{3}=\left\{k\left(f_{1},g_{1},f_{2}\right),k\left(f_{2},g_{2},f_{3}\right)⟹k\left(f_{1},\left(g_{1},g_{2}\right),f_{3}\right)\right\}. \end{array}$

In this definition, *F*_1_ is the set of relationships between processing objects and devices. *F*_2_ is the set of relationships between processing object properties. *F*_3_ is the set of relationships between equipment parameters. *P*_1_ and *P*_2_ are the basic structure sets of processing objects and processing devices, respectively. Using the rules in *P*_3_, the chain of relationships from raw materials of TCM to products can be obtained. If semiproduct *f*_2_ is made from raw material, *f*_1_ through device *g*_1_ and product *f*_3_ can be made from semiproduct *f*_2_ through device *g*_2_, the production line *f*_1_⟶*g*_1_⟶*g*_2_⟶*f*_3_ can be obtained according to the rules in *P*_3_. *S* stands for the initial condition in the system.

TMIM has advanced production concepts of personalized customization, flexible equipment combination, and information network transmission. It is a general intelligent manufacturing paradigm, which can be used to simulate hierarchical structure of complex systems and guide construction of intelligent systems.

### 3.3. The Design of Data Flow Logic Framework Based on TMIM

In TCM-ISP, data transfer is at the core of platform system construction, which runs throughout the platform system. Under the guidance of TMIM, this paper analyzed the logical framework of data flow in detail to lay the foundation for scheme design of Chinese medicines intelligent service platform.

On the basic of TMIM, a quadruple *Q*=(*V*, *F*, *P*, *S*) can also represent the logical framework of data flow of TCM-ISP:

1. *V*=*V*_1_ ∪ *V*_2_ ∪ *V*_3_ ∪ *V*_4_ ∪ *V*_5_.
2. $\begin{array}{c} F=\left\{f_{1},g_{1}\right\},\\ f_{1}=\left\{f_{1}\left(b,c,d,e\right),b\in V_{2},c\in V_{3},d\in V_{4},e\in V_{5}\right\},\\ g_{1}=\left\{g_{1}\left(a_{1},a_{2},\ldots \ldots ,a_{n}\right),\;a_{i}\in E\left(V_{2}\cup V_{3}\cup V_{4}\cup V_{5},f_{1}\right)\right\}. \end{array}$
3. *P*={*k*_1_(*a*_1_, *b*_1_, *a*_2_), *k*_2_(*a*_2_, *c*_1_, *a*_3_)⟶*k*_3_(*a*_1_, *b*_1_, *c*_1_, *a*_3_)}.
4. *S* ∈ (*s*_1_, *s*_2_, *s*_3_,…*s*_*m*_),  *s*_*i*_ ∈ *E*(*V*_2_ ∪ *V*_3_ ∪ *V*_4_ ∪ *V*_5_, *f*_1_).

In the above definition, *V* refers to the basic object in TCM-ISP, that is to say, the collection of data information and work units in the platform system. *V*_1_: the set of data in the system. *V*_2_: data acquisition unit, a collection of sensory devices. *V*_3_: display unit, a collection of data presentation forms. *V*_4_: data processing unit, a collection of storage, control, and algorithms. *V*_5_: control unit, a collection of application devices.

*F* is the basic structure of workflow of TCM-ISP. *f*_1_ is the basic combination pattern of work units in TCM-ISP. *G*_1_ refers to the transfer mode of the data information in flexible combined work unit. Each workflow consists of *N* elements “*a*” in which any “*a*_*i*_” belongs to the set of entities formed by combination of data information elements and work units.

*P* represents the rule required for inference and is the main relation on which the combination of work units relays, that is to say, using the transmission rules of data information to infer the combination mode of working units. Moreover, *S* stands for the initial condition, which is composed of *M* elements “*S*.” Under the guidance of TMIM, the combination patterns of data information and work unit are designed to build the logical structure of the data flow based on the rule set *P* and data information.

### 3.4. Overall Structural Framework of Chinese Medicines Intelligent Service Platform

The overall structural framework of TCM-ISP was built through the data flow logic framework with data of overall platform system as the core. As shown in Figure 3, the platform system consists of three units, including data acquisition unit, central control unit, and device unit. Within TCM-ISP, data acquisition unit is a collection of sensory devices that are responsible for data acquisition; device unit is a collection of application devices in the platform system. In addition, central control unit is a service window for data display and data processing, responsible for data display, data storage, remote control, user management, data interaction, and other service functions. In overall architecture of the platform, each functional component and application are relatively independent, which reduces the coupling of the platform and makes the platform have good scalability and cross-platform.

## 4. Technology Implementation Roadmap of Chinese Medicines Intelligent Service Platform

TCM-ISP focused on the communication of data information in different units, aiming to provide users with a convenient and easy-to-operate comprehensive service platform. According to the overall structure of TCM-ISP, platform system contains two parts: one is the server side platform; the other is the monitoring point. The monitoring point that is composed of sensory unit, equipment unit, and embedded equipment can carry out data acquisition, data conversion, data transmission, command reception, and equipment feedback. The server side platform consists of data display, data storage, and data processing units and it has a man-machine interface, which can read, store, process, display, and issue commands.

In the following section, we will describe the hardware structure diagram of monitoring point and the software technology diagram of server side platform.

### 4.1. Hardware Structure of Monitoring Points

In Chinese medicines intelligent service system (TCM-ISP), each monitoring point can process the collected data from sensors in a definite way and communicate with the service platform through API. According to logical framework of data flow, the monitoring point is a collection of data collection units and control units, which are responsible for collecting data and flexible scheduling of equipment, etc. In this research, we developed networked monitor nodes using Raspberry Pi and Arduino.

As shown in Figure 4, in order to ensure the flexible configuration of monitoring points, as well as the scalability of sensors in monitoring points, we adopted the modular design idea of separate Raspberry Pi and sensor. At the same time, we proposed to use CH340 USB-TTL and TTL-RS485 to design a unified interface between boards with supporting hot-plugging mode. In the above way, when collecting new data information due to different requirements, the developer only needs to develop a new sensor board according to the unified plug-in interface, without completely redesigning monitoring points as a whole. The applied hardware devices in monitoring points include Raspberry Pi Zero W, various sensors, Arduino Nano, CH340 USB-TTL, and TTL-RS485.

As a microcontroller, Raspberry Pi is the carrier of Arduino Nano and various sensors, which not only reads and controls the lower data but also interacts with the upper service interface. Raspberry Pi is a low-cost minicomputer, among which Raspberry Pi Zero which is the more suitable in the Raspberry Pi family [19–21]. Raspberry Pi can run a variety of systems such as Linux and Windows systems. It has a built-in Wi-Fi/BT wireless chip that greatly enhances communication capabilities. Moreover, the Raspberry Pi has a variety of interface peripherals, including USB port, SD card, and expandable GPIO pins [22, 23]. As a result, the Raspberry Pi can process, store, and upload data collected by multiple sensors.

Connecting Arduino with sensor to design the sensor module. Arduino is a convenient and flexible open source hardware with characteristics of cross-platform, simplicity-clarity, and openness [24, 25]. Arduino Nano contains two main parts: hardware and software, which can be plugged directly into the breadboard. Hardware part is the link circuit of various Arduino circuit boards. Software refers to a program development environment in the computer provided by Arduino IDE. Similarly, Arduino Nano can not only connect with a variety of sensors to sense environment but also control the corresponding devices to provide feedback and influence for the environment [26, 27].

With regard to signal conversion, we adopted TTL-RS485 and CH340G adapters. TTL-RS485 is a converter that can realize mutual conversion between TTL signal and RS485 bus, which can guarantee the synchronization of signal data and direct access to the network. Therefore, TTL-RS485 bus connection and self-developed communication protocol were selected to realize signal conversion and complete the communication between systems. CH340G is a USB bus adapter chip that provides a MODEM contact signal for USB to serial port. It is beneficial for the platform to expand asynchronous serial port, thus ensuring flexible configuration of monitoring points and normal transmission of data stream.

### 4.2. Software Technology Roadmap of Server Side Platform

In TCM-ISP, the server side platform had human-machine interface for providing services, which was designed on the foundation of analyzing user requirements and data flow logic framework. It provided the user with a service window with multiple functions such as data storage, processing, and command distribution.

Software technology roadmap is shown in Figure 5. The platform adopted a typical browser/server structure, in which data transfer is the core, as well as monitoring points are both data collection point and device control point. The server side platform consists of three parts: database, web service, and server side. Database is mainly responsible for storage of data. Considering MySQL is an open source relational database system and its advantages, MySQL, along with PHP and Apache, can provide a good development environment to build back-end databases. Web service provides multiple services such as data display, remote control, user management, and data interaction functions. In web application development, we chose PHP scripting language as the main development language of dynamic application.

At the same time, HTML, CSS, and JavaScript were used to establish the front-end interactive interface, in which HTML was used to mark up and design web pages, and JavaScript was used for client-side scripting to support dynamic displays and interactive user interfaces. Web back-end used timer to request data from the data center at regular intervals. Web service interface adopted a friendly graphical interface that contains login interface, real-time monitoring interface, history query interface, data chart interface, algorithm selection interface, and device management interface. Users can access sensor data or perform configuration and management of deployed detection points via terminal or local area network.

## 5. Test of Chinese Medicines Intelligent Service Platform

Based on analysis of user requirements and overall construction plan of the platform, we completed the construction of TCM-ISP. The platform homepage, shown in Figure 6, provided four functions of user management, monitoring point management, device management, and sensor management. On this basis, we tested the function of platform to ensure its feasibility.

### 5.1. User Management

The user completed registration in the platform, and when logged in, the user clicks on the user center to enter platform interface. As shown in Figure 7, the TCM-ISP showed all registered users in the user management module, which contains two categories of ordinary users and administrators. Administrators can edit, add or delete and set user permissions, etc.

### 5.2. Management of Devices and Sensors

The initial interface of device management is shown in Figure 8. Device management module can add, edit, and delete sensors and devices according to requirements. When logging into the interface, the user can see all the devices set up in the monitoring point. The platform provided managers with flexible and scalable sensor access points. When a new device is added to the monitoring point, the user can click “Add” button on the device management page to fill in the device information to complete the flexible configuration.

### 5.3. Operation of Data Information in TCM-ISP

As for data acquisition, processing, and device control aspects in TCM-ISP, we took the temperature-humidity sensor module and relay module as an example to test the platform system from data flow process to the device feedback. The data acquisition module consists of a combination of temperature-humidity sensor, switching devices, Raspberry Pi Zero W, and Arduino Nano hardware devices. Platform data upload path contains the following steps: (1) sensors sense the surrounding environment to convert a physical signal into an electrical signal. (2) Using Arduino Nano's A/D conversion function to digitize the sensor signal. (3) After getting sensor data, Arduino Nano sends the data code to Raspberry Pi using the serial port, and Raspberry Pi Zero W communicates with the server via TCP protocol to store data into MySQL database.

In data display process, firstly, the user sends a request on the web interface; secondly, the above request instruction accesses backstage database through PHP; finally, search result based on request instruction feeds back to interface for data display. The platform can realize both real-time display of data and review of historical data, in which data are presented in the form of statistical curves or data tables. Meanwhile, you can view data changes within the set time range. Figures 9 and 10 show the real-time temperature-humidity data of environment and the ambient temperature-humidity data read by the back-end server, respectively.

Figures 11 and 12 show the line graphs of historical data of ambient temperature and humidity, respectively.

Regarding the calculation and processing of data, the platform provided a window for flexible data processing, in which users can add their own algorithms as needed. The data processing interface is shown in Figure 13.

### 5.4. Control of Application Equipment

Users can set threshold conditions in trigger interface according to the type of monitoring data. When meeting trigger conditions, the platform can realize the flexible, intelligent, and networked regulation of equipment through relays. As shown in Figure 14, this is the setting interface of trigger condition. In addition, users can also send open or close commands to the server by clicking on the switch button in the service interface. Further, when receiving command, the server sends a command to the relay to complete remote networked control of devices. Simultaneously, the operation status of the application device was displayed in the service interface as shown in Figure 15.

According to the functions of the platform, we successfully finished the registration, login, and management of user and arrangement of monitoring points as well as management of sensors and equipment. Moreover, we took the temperature-humidity sensor module and relay module as an example to verify the feasibility of TCM-ISP operation. The result shows that TCM-ISP can not only realize the integration, real-time transmission, and display of data information but also well accomplish remote intelligent-flexible control of equipment and carry out flexible scheduling, intelligent self-regulation, and network transmission according to the requirements of users. It is of great significance to solve the current difficulties of low informatization and intelligence in Chinese medicines industry and promote the development of intelligent manufacturing in Chinese medicines industry.

## 6. Discussion

### 6.1. Advantages of Theoretical Model of Intelligent Manufacturing of Chinese Medicines

Theoretical model of intelligent manufacturing of Chinese medicines (TMIM) was mainly proposed to address the lack of theoretical guidance in the development process of intelligent manufacturing of Chinese medicines. TMIM's core features are the pursuit of intelligence, networking, and flexibility with the solid theoretical foundation-entity grammar system and support of modern science technology [17, 18]. A generic intelligent manufacturing paradigm, TMIM, can simulate complex structures in intelligent systems and especially guide the construction of intelligent systems. Therefore, we use TMIM to simulate the data framework system of the intelligent platform to depict the combination and transmission of data and individual units in detail and objectively, which is beneficial to understand the logical relationship of platform system and later digital programming.

### 6.2. Construction of Intelligent Service Platform for Traditional Chinese Medicines

In order to realize real-time monitoring, information communication, and intelligent scheduling of equipment in whole TCM's industry chain and to promote modernization of Chinese medicines industry, in this paper, we designed the intelligent service platform for Chinese medicines (TCM-ISP).

Data flow is the transfer of data between units of the platform. In the early stage of building TCM-ISP, data flow framework system of the platform was established on the basic of TMIM. Although the form of data in each link of TCM is different, the rules of data transmission are the same in each link [28]. The construction of a data flow framework system is conducive to clarifying the data transmission rules between units and sorting out the logical relationship between the data operation of each unit to establish TCM-ISP.

The successful establishment of TCM-ISP cannot be achieved without support of modern science technology. New-generation information technology ensures the networked and intelligent operation of TCM-ISP such as wireless communication, cloud computing, and sensors [15, 29]. However, due to different sensing devices and communication protocols of each link, it is difficult for the platform system to achieve unified scheduling or complete flexible configuration according to demand. To solve the problem of flexible configuration or scheduling, this paper proposes a modular design idea of separate Raspberry Pi and sensor modules. On the premise of modular design concept, CH340, USB-TTL, and TTL-RS485 were used to design a unified interface between boards, supporting mode of hot plugging. In the hot-plugging mode, it is easy to develop new sensor boards without the requirement to redesign the entire monitoring front-end.

### 6.3. Features of the Chinese Medicines Intelligent Service Platform

The Chinese medicines intelligent service platform (TCM-ISP) was established based on the theoretical model of intelligent manufacturing of traditional Chinese medicines (TMIM). With the purpose of serving the public, it also pursues personalized service, flexible configuration, and intelligent collaboration. TCM-ISP is a dynamic mobile universal service platform in which users can interact with the web application on the LAN or log in to the web interface from any terminal on the Internet to access. Not only can managers easily deploy multimonitoring applications on TCM-ISP but they can also add sensors and application devices according to requirements. TCM-ISP effectively overcomes the main drawbacks of the existing platform, namely, the limitation of services, static configuration, which makes it difficult to adapt to the diversity, integration, interaction, and overall planning of information in each links of the Chinese medicines industry chain. In addition, the monitoring points of the platform adopt the mode of modular separation and hot plug-in unified interface, which provides users with flexible and extensible sensor access points.

## 7. Conclusion

In this paper, an easy-to-operate, extensible, and comprehensive Chinese medicines intelligent platform (TCM-ISP) with characteristics of flexibility, versatility, and individuation was constructed under the guidance of theoretical model of intelligent manufacturing of Chinese medicines. TCM-ISP is a comprehensive intelligent service platform, which breaks through limitations of existing platforms that were more designed for specific segments or provide a single service. TCM-ISP can not only successfully realize the integration, real-time transmission, and display of data information but also well accomplish remote intelligent-flexible control of equipment and allow flexible configuration and expansion of sensors and devices according to the needs of each link in TCM's industry chain. It is of great practical significance to the pursuit of intelligent manufacturing of Chinese medicines and the promotion of modernization of Chinese medicines industry.

## Figures and Tables

**Figure 1:** Chinese medicines intelligent service platform systems.

**Figure 2:** Functional framework of Chinese medicines intelligent service platform.

**Figure 3:** Overall structural of Chinese medicines intelligent service platform.

**Figure 4:** Hardware structure diagram of monitoring points.

**Figure 5:** Software technology roadmap of server side platform.

**Figure 6:** Homepage of Chinese medicines intelligent service platform.

**Figure 7:** The interface of user management.

**Figure 8:** Management interface of devices and sensors.

**Figure 9:** Real-time data of temperature-humidity.

**Figure 10:** Ambient data of temperature-humidity.

**Figure 11:** Data graph of ambient temperature.

**Figure 12:** Data graph of ambient humidity.

**Figure 13:** Processing interface of data in TCM-ISP.

**Figure 14:** The setting interface of trigger.

**Figure 15:** The display interface of device status.

## Data Availability

This article does not deal with experimental data and data analysis; the article deals with the establishment of the TCM-ISP service platform. The authors did not get permission to share the data.
